This article has been retracted.

# Clinical Application of the Classical Theory of Traditional Chinese Medicine in Diabetic Nephropathy

**DOI:** 10.1155/2022/4066385

**Published:** 2022-04-20

**Authors:** Jintong Pan, Huihui Li, Junhua Shi

**Affiliations:** ^1^Hubei Province Hospital of Traditional Chinese Medicine, Nephropathy, China; ^2^Guangzhou Weimi Biological Technology Company, China

## Abstract

**Objective:**

To explore the clinical application of the classical theory of traditional Chinese medicine (TCM) in diabetic nephropathy (DN).

**Methods:**

A total of 100 patients with DN treated in our hospital from May 2019 to June 2021 were included. The patients were randomly assigned to the control group and the study group. The control group received routine treatment, and the study group was treated with the classical theory of TCM. The efficacy, TCM syndrome score, urine proteinuria (UTP), urine albumin-creatinine ratio (UACR), plasma albumin (ALB), hemoglobin A1c (HbA1C), fasting blood glucose (FBG), blood urea nitrogen (BUN), creatinine (Cr), and treatment safety were compared between the two groups.

**Results:**

In comparison to the curative effect, the study group was significantly effective in 34 cases, effective in 12 cases, and ineffective in 4 cases, and the effective rate was 92.00%; the control group was significantly effective in 16 cases, effective in 18 cases, and ineffective in 16 cases, and the effective rate was 68.00%. The effective rate in the study group was higher compared to the control (*P* < 0.05). In comparison to the TCM syndrome scores, there exhibited no significant difference before treatment (*P* > 0.05), but after treatment, the TCM syndrome scores of the two groups decreased, and the TCM syndrome scores of the study group were lower compared to the control at 6 weeks, 12 weeks, 24 weeks, and 36 weeks of treatment (*P* < 0.05). There exhibited no significant difference in the indexes of UTP and UACR before treatment, but the indexes of UTP and UACR in the two groups decreased after treatment, and the indexes of UTP and UACR in the study group were lower compared to the control at 6 and 12 weeks after treatment. There was no significant difference in the indexes of ALB, HbA1C, and FBG before treatment, but after treatment, the indexes of ALB increased, the indexes of HbA1C and FBG decreased in both groups, and the indexes of HbA1C and FBG i4n the study group were lower compared to the control, while the index of ALB in the study group was higher. The indexes of BUN and Cr were compared, and there was no significant difference before treatment, but after treatment, the indexes of BUN and Cr in the two groups decreased, and the indexes of BUN and Cr in the study group were lower compared to the control (*P* < 0.05). In terms of the treatment safety of the two groups, there was no abnormality in blood, urine, stool routine, and liver and kidney function examination in the study group. No obvious adverse reactions were found in all patients. There were 1 case of abnormal liver function and 2 cases of rash in the control group, and there exhibited no significant difference (*P* > 0.05).

**Conclusion:**

Under the guidance of classical theory, the optimization scheme of comprehensive treatment of TCM may improve renal function by improving metabolic disorders, vascular lesions, neurotrophic disorders, antioxidant stress, and other ways to repair nerve injury, improving the changes of TCM syndromes, signs, and indicators of patients, and delay the progress of DN.

## 1. Introduction

Diabetic nephropathy (DN) is one of the most common and serious chronic complications of diabetes mellitus (DM), which is systemic microangiopathy by DM, and it is also the main cause of death in patients with DM [1]. The main manifestations are varying degrees of proteinuria and progressive decline of renal function. According to the results of the survey, by 2016, the global prevalence rate of DM is about 9.3%, while the epidemiological survey in China shows that the incidence of DM is 10.4% [2]. About 116 million people in China are suffering from it [2], and about 40% of these people have been complicated with DN [3]. If we do not take a positive attitude and timely intervention, and DN will continue to progress, renal function will continue to decline and soon develop into end-stage renal disease (ESRD), resulting in irreversible kidney damage, so that the quality of life of patients has been seriously affected. At present, DN has become the first cause of ESRD [3]. We should pay enough attention to early detection and active intervention to delay the progress of the disease as much as possible [4]. The pathogenesis of DN is complicated, and there is no unified conclusion at present. Experts and scholars believe that it is related to the alterations of hemodynamics, nonenzymatic glycosylation of protein, increase of polyol channel activity, change of glomerular filtration barrier, inflammatory factors, oxidative stress, heredity, and so on [5–7]. At present, there is a lack of effective specific treatment for DN, modern treatment mainly through diet control and other primary diseases of drug intervention, to reduce kidney damage as much as possible, but the effect is very little [8]. Therefore, finding an effective method of prevention and treatment of DN in traditional medicine has become one of the important missions.

DN belongs to the diagnostic name of modern medicine, referring to the classical ancient books of TCM, and there is no detailed record of DN, but according to its clinical symptoms, signs, and trends of disease development, it can be classified into the categories of “eliminating thirst,” “edema,” “turbid urine,” “virtual fatigue,” “Guange,” and so on [3]. With the deepening of physicians' understanding of this disease, the work related to this disease is gradually increasing. According to Professor Lu Renhe's book “*Diagnosis and Treatment of Diabetes and Its Complications of Traditional Chinese and Western Medicine*” [9], the symptoms such as edema, increase of urine foam, nausea and vomiting, skin itching, oliguria, and anuria that gradually appear in DM are summarized as “Antithirst Nephropathy.” DM belongs to the syndrome of yin deficiency and internal heat, the course of the disease is long, it is lingering and does not heal, and kidney injury occurs, which consumes vital qi, dryness, and heat, and further consumes qi, resulting in the syndrome of deficiency of both qi and yin; the patient's deficiency of vital qi, abnormal operation of qi, inability to promote, leading to internal stagnation of tangible pathogens such as phlegm, water, and dampness, further blocking qi, heat, and dampness for a long time, the evil gel of dampness and heat, making the disease more lingering and difficult to recover [10]. When a long-term illness enters the collaterals, there is the appearance of internal stagnation of blood stasis. Therefore, most DN belongs to deficiency and excess. According to the characteristics of etiology and pathogenesis, it is proposed that the treatment of DN should be based on replenishing qi and nourishing yin, as well as removing dampness and activating blood circulation. For many years, when applying the diagnosis and treatment plan of the State Administration of TCM, we found that the scheme has some defects, such as narrow syndrome coverage, that cannot fully reflect the complicated clinical changes, poor curative effects, and so on. It is far from meeting clinical needs [10]. Under the guidance of the policy of “reading classics, doing clinical work, and following famous teachers” of the State Administration of TCM, we apply the classical theory to the clinic, adopt syndrome differentiation of the six meridians, add and subtract treatment with the meridian prescription as the base, and further enrich and improve the characteristic therapy of TCM. Through several years of clinical observation, practice, and summary, we have formed a set of effective, simple, and convenient optimization schemes with outstanding characteristics of TCM and achieved satisfactory results in a clinic.

## 2. Patients and Methods

### 2.1. General Information

A total of 100 patients with DN treated in our hospital from May 2019 to June 2021 were included. The patients were randomly divided into the control group and study group. In the control group, the age was 43-85 years old, with an average of 58.77 ± 2.67 years, including 27 males and 23 females, while in the study group, the age was 44-86 years old, with an average of 58.67 ± 2.55 years, including 24 males and 26 females. There was no statistical significance in the general data of the two groups. This study was approved by the Medical Ethics Association of our hospital, and all patients signed informed consent.

The diagnostic criteria of western medicine are as follows: refer to the diagnostic criteria of DN in the guidelines for diagnosis and treatment of DN [11].

The standard of syndrome differentiation of TCM is as follows: the treatment group adopted the syndrome differentiation of six meridians in Treatise on Febrile Diseases: Sun, Yangming, Shaoyang, Taiyin, Shaoyin, and Jueyin. The control group referred to the diagnosis and treatment scheme of arthralgia syndrome (DN) of arthralgia syndrome in 22 specialties and 95 diseases issued by the State Administration of TCM in 2010. Thirst arthralgia's clinical common syndromes are as follows: (1) qi deficiency and blood stasis syndrome; (2) cold coagulation and blood stasis syndrome; (3) yin deficiency and blood stasis syndrome; (4) phlegm and blood stasis blocking collaterals: the limbs are numb, often fixed, such as stepping on cotton, sleepy limbs, head weight such as wrapping, dizziness, obesity, sticky mouth, stuffy chest, abdominal distension and discomfort, and sticky stools; (5) deficiency of liver and kidney syndrome: weakness of limbs, muscle atrophy, even impotence, sore waist and knees, impotence, loose teeth shaking, dizziness and tinnitus, light tongue, little or no fur, and weak pulse; and (6) kidney deficiency and blood stasis syndrome.

The inclusion criteria were as follows: (1) those who met the above diagnostic criteria of DN; (2) older than 18 years old; (3) less fluctuating and well-controlled blood glucose in the last 2 months; (4) conscious and free from mental disorders; (5) no treatment of DN within 3 months before treatment; and (6) voluntarily participated in this trial and signed an informed consent form.

The exclusion criteria are as follows: (1) patients with other serious acute and chronic complications of diabetes (such as proliferative retinitis, the disappearance of pulsation of the dorsalis pedis artery or posterior tibial artery); (2) severe heart, brain, kidney disease, malignant tumor, chronic alcoholism, etc.; (3) severe mental stimulation, severe trauma, surgery, and other stress states; (4) long-term bedridden; (5) pregnant and lactating women; (6) long-term alcoholism; (7) mental or psychological disorders; (8) limb deformities, trauma, or edema; and (9) people with allergic constitution and allergies to a variety of drugs.

### 2.2. Treatment Methods

Both groups were given basic treatment of diabetes: diabetes education, diet, exercise, oral hypoglycemic drugs and/or insulin, blood pressure control, lipid regulation, and so on. Use vasodilators, nutritional nerve agents, antiplatelet aggregators, aldose reductase inhibitors, gangliosides, antioxidants, circulatory agents, and other drugs.

The control group adopted the diagnosis and treatment scheme of “eliminating thirst nephropathy” issued by the State Administration of TCM: (1) qi deficiency and blood stasis syndrome: treated with tonifying qi and activating blood, removing blood stasis, and dredging collaterals, plus or minus Buyang Huanwu decoction; (2) cold coagulation and blood stasis syndrome: treated with warming meridians and dispelling cold, dredging collaterals, and relieving pain, plus or minus Danggui Sini decoction; (3) yin deficiency and blood stasis syndrome: treated with nourishing yin and activating blood, tendon priority, and Shaoyao Gancao decoction combined with Siwu decoction; (4) syndrome of phlegm and blood stasis blocking collaterals: treated by resolving phlegm and promoting blood circulation, promoting arthralgia, and dredging collaterals, referring to Mi Fuling pills combined with Huangqi Guizhi Wuwu decoction; (5) liver and kidney deficiency syndrome: treated with nourishing liver and kidney, filling pulp, and filling meat, plus or minus Zhuanggu pills; (6) kidney deficiency and blood stasis syndrome: it is treated by tonifying the kidney and activating blood, and deer antler prescription is added or subtracted. Acupuncture and moxibustion therapy are as follows: specifically combined with the suggestion of acupuncture and moxibustion consultation doctors, acupuncture and moxibustion doctors should carry out the treatment, and choose different treatment methods such as body acupuncture, ear acupuncture, and electroacupuncture according to the needs of the disease. Massage therapy is as follows: choose according to the needs of the disease.

The research group adopted the syndrome differentiation of six meridians: (1) cold and dampness blocked the sun meridians: upper and lower limbs or back numbness, cold sensation, muscle soreness, easy to catch a cold, reddish tongue, thin white coating, and pulse floating string. It is treated by dispelling cold and dehumidification, warming channels, and dredging collaterals, and adding and subtracting Huangqi Guizhi Wuwu decoction and Mahuang decoction; (2) cold and dampness blocking Shaoyang meridians: numbness, pain, cold on the outside of the limbs, bitter mouth in the morning, stuffy chest, poor stomach, light red tongue, thin white fur, and fine pulse. Treat the meridians of warming Shaoyang and add or subtract Chaihu Guizhi decoction; (3) cold and dampness blocking Jueyin meridian: numbness, cold, and ant sensation on the inside of thigh and leg, accompanied by parietal pain, drooling, loose stool, reddish tongue, thin white fur, sinking pulse. To warm the liver and warm the meridian, remove dampness and dissipate cold and add and subtract Angelica Sini plus Evodia and ginger decoction; (4) Shaoyin deficiency and cold stagnation: cold and pain at the ends of the extremities, decreased temperature, aggravated cold, heavy at night, often difficult to fall asleep, heavy and tired, long urine, loose stool, dark lips and green tongue, fat tongue, slippery fur, and weak pulse. Treat with warming yang and replenishing qi, dispelling cold and relieving pain, give aconite soup, *Astragalus* cinnamon twig Wuwu decoction, and Mahuang Fuzi Asarum decoction to add or subtract; (5) the disease of Shaoyin, Yang, and Ming: it shows viscera heat, meridian cold, limb pain, numbness, cold, bad breath, burning heart and chest, mouth sores, yellow urine, dry stool, red tongue, fat tongue, white greasy or yellow greasy fur, and slippery pulse for several feet. Treat warm meridians and collaterals, cold and clear viscera heat, add and subtract aconite decoction and rhubarb lian Xiexin decoction; (6) deficiency of Taiyin, Yang Qi depression: fever of limbs or muscle surface, body like fire, cauterization of hands, light red tongue, thin white fur, and deep and thin pulse. When the fire is depressed, it is added or subtracted by Shengyang Sanhuo decoction. With the characteristic therapy of TCM, TCM foot bath is prescribed (raw ephedra, transparent bone grass, cassia twig, chicken blood vine, stretching muscle grass, Chuanxiong, moxa leaf, safflower, and sappan wood), water frying 800°C, keep water temperature 40°C, foot bath 20-30 min, 1-2 times a day. TCM iontophoresis therapy (peach kernel, Angelica sinensis, Rhizoma Drynariae, Radix Asarum, Rhizoma Corydalis, Radix Polygoni Multiflori, Radix Polygoni Multiflori, Radix safflower, Radix Achyranthes bidentata, mulberry twig, etc.), decocted and concentrated, and the solution was treated by medium frequency iontophoresis instrument, once a day. Acupuncture therapy is as follows: according to the principle of “Sheng is purging, deficiency is tonifying, heat is disease, cold is staying, and sinking is moxibustion,” the treatment is classified into different types. Moxibustion and acupoint application is as follows: Geguning pill cake moxibustion or acupoint application at Sanli, Quchi, Waiguan, Hegu, Zusanli, Xuehai, Yanglingquan, Yongquan and other acupoints, once a day. Acupoint injection is as follows: vitamin B1 and mecobalamin were injected at Zusanli and Quchi, once a day. Characteristic nursing of TCM is as follows: including health guidance, condition observation (symptoms, concomitant symptoms, limb appearance, etc.), general nursing, diet nursing, medication nursing, syndrome differentiation nursing, health care of TCM, etc.

### 2.3. Observation Index

#### 2.3.1. Curative Effect Evaluation

The curative effect of TCM syndrome is as follows: it is judged according to the scoring method of TCM syndrome. It was formulated according to the guiding principles of Clinical Research of New drugs of TCM [12] (2002 trial version). Efficacy index = (pre − treatment score − post − treatment score)/pre − treatment score × 100%. Note: the calculation formula (nimodipine method) clinical recovery: TCM symptoms and signs disappear or basically disappear, syndrome scores are reduced by ≥90%; effective: TCM symptoms and signs are improved, and syndrome scores are reduced by ≥70%; effective: TCM symptoms and signs are improved, and syndrome scores are reduced by ≥30%; ineffective: TCM symptoms and signs are not significantly improved or even aggravated, and syndrome scores are reduced by less than 30%. Effective rate of treatment = markedly effective rate + effective rate.

#### 2.3.2. TCM Syndrome Integral

TCM syndrome score is as follows: formulated with reference to the guiding principles of Clinical Research on New drugs of TCM (2002 trial version). They were assigned into mild (2 points), moderate (4 points), and severe (6 points). The TCM syndrome scores of the two groups before treatment, 6 weeks, 12 weeks, 24 weeks, and 36 weeks were counted.

#### 2.3.3. Serum Index Detection

In the early morning fasting state, after EDTA anticoagulation treatment, 3000 rpm, centrifugation 10 min, the upper serum was frozen at -80°C to be tested. The levels of urine proteinuria (UTP), urine albumin-creatinine ratio (UACR), plasma albumin (ALB), hemoglobin A1C (HbA1C), fasting blood glucose (FBG), blood urea nitrogen (BUN), and creatinine (Cr) in serum were detected by enzyme-linked immunosorbent assay (ELISA). All the kits are purchased from the Redd Company of the United States and operate strictly in accordance with the standards of the instructions. The intrabatch differences are less than 10%, and the interbatch differences are less than 15%. UTP and UACR indexes were collected before treatment and 6 weeks and 12 weeks after treatment. The indexes of ALB, HbA1C, FBG, BUN, and Cr were collected before and after treatment.

#### 2.3.4. Safety Index

The blood, urine, stool routine, and liver and kidney function tests were improved in both groups, and the incidence of adverse reactions in the two groups was calculated.

#### 2.3.5. Statistical Analysis

The data were statistically processed by the SPSS21.0 software, the counting data were tested by the chi-square test, and the measurement data were expressed in $\bar{x}\pm s$. The comparison between groups was first tested for normality and homogeneity of variance, and the single-factor analysis of variance and group *t*-test was employed for those who satisfied normality and homogeneity of variance. For those who did not satisfy the homogeneity of normality and variance, the Kruskal-Wallis *H* test of multiple independent samples in the nonparametric test was employed for comparison among the three groups, and the rank-sum test of the paired design data of the two related samples in the nonparametric test was employed for intragroup comparison. The rank-sum test was employed for the grade data, and the difference was statistically significant (*P* < 0.05). A *P* value less than 0.01 was viewed as highly statistically significant.

## 3. Results

### 3.1. Comparison of Curative Effect

First of all, we compared the curative effects of the two groups: the study group was significantly effective in 34 cases, effective in 12 cases, and ineffective in 4 cases, and the effective rate was 92.00%; the control group was significantly effective in 16 cases, effective in 18 cases, and ineffective in 16 cases, and the effective rate was 68.00%. The effective rate in the study group was higher compared to the control (*P* < 0.001). All the data results are shown in Table 1.

### 3.2. Comparison of Syndrome Scores of TCM

Secondly, we compared the TCM syndrome scores of the two groups. Before treatment, there was no significant difference (*P* > 0.05). The TCM syndrome scores of the study group were lower compared to the control at 6 weeks, 12 weeks, 24 weeks, and 36 weeks of treatment (*P* < 0.05). All the data results are shown in Table 2.

### 3.3. UPT and UACR Index Comparison

Next, we compared the indexes of UTP and UACR, and there was no significant difference before treatment; however, the indexes of UTP and UACR decreased in both groups after treatment. The UTP and UACR indexes in the study group were lower compared to the control at 6 and 12 weeks after treatment (*P* < 0.05). All the data results are shown in Figure 1.

### 3.4. ALB, HbA1C, and FBG Index Comparison

Then, we compared the indexes of ALB, HbA1C, and FBG, and there was no significant difference before treatment, but after treatment, the indexes of ALB increased, and the indexes of HbA1C and FBG decreased in the two groups. The indexes of HbA1C and FBG in the study group were lower compared to those in the control, while the ALB index was higher (*P* < 0.05). All the data results are shown in Figure 2.

### 3.5. BUN and Cr Index Comparison

Next, we compared the indexes of BUN and Cr, and there was no significant difference before treatment. After treatment, the indexes of BUN and Cr in the two groups decreased, and the indexes of BUN and Cr in the study group were lower compared to the control. All the data results are shown in Figure 3.

### 3.6. Comparison of Safety Evaluation

Finally, we compared the treatment safety of the two groups, and no abnormality was found in blood, urine, stool routine, and liver and kidney function tests in the study group. No obvious adverse reactions were found in all patients. There were 1 case of abnormal liver function and 2 cases of rash in the control group, and there was no significant difference between the two groups (*P* > 0.05).

## 4. Discussion

TCM syndrome differentiation of DN is the name of pseudodiabetic kidney disease in TCM, focusing on the essence of pathological changes and the relationship between evil and good at a specific stage of diabetes, to understand the etiology, disease location, disease situation, pathogenesis, and nature, in order to achieve the purpose of new balance treatment [13]. Accurate syndrome differentiation is to determine the nature, essence, syndrome type, and outcome of the disease and take the syndrome as the center of the unique operation [5]. DN in TCM and its clinical practice are attributed to “diabetes,” which belongs to the category of complications and belongs to the category of the syndrome such as elimination of diabetes, fat and noble people, turbid urine, and edema [13]. The characteristics of mutual root and intercommunication of the lesions determine that the prognosis is difficult to be optimistic about. The nature, characteristics, mechanism, classification, and evolution outcome of the lesions depend on the occurrence of different complications, and diabetic kidney disease is one of the serious complications. Doctors of later generations have their own expositions on the blank part of the contents of eliminating thirst in Internal Classic of Medicine, Jin Jing, and Internal Medicine of TCM [14–16]. The Theory of Sugar and Collateral Miscellaneous Diseases points out the pattern of uncertain complications of diabetes: the regular characteristics, guiding ideology, and theoretical basis of “the disease enters the collaterals for a long time, from collaterals to miscellaneous collaterals.” And Ye Tianshi's concluded that “long illness enters collaterals.” Based on the ancient and modern theory, the operation or permission for predicting the occurrence of different complications in different periods of time is explored from the methodology of five stages: occult period, early stage, middle stage, and late stage. TCM syndrome differentiation of DN is the name of pseudodiabetic kidney disease in TCM, focusing on the essence of pathological changes and the relationship between evil and good at a specific stage of diabetes, to understand the etiology, disease location, disease situation, pathogenesis, and nature, in order to achieve the purpose of syndrome differentiation from the new balance theory [17].

Taking the macroscopic, holistic concept and dialectical thinking as the guiding ideology and taking the syndrome characteristics of diabetic kidney disease as the guide, TCM guides the reasoning and analysis of the comprehensive contents of etiology and pathogenesis [18]. Accurate syndrome differentiation is to determine the nature, essence, syndrome type and outcome of the disease, and the unique operation centered on syndrome [19]. Neijing highly generalizes the theoretical basis of diabetes: “overflow,” “elimination,” and “diabetes” belong to the category of diabetes classification, and diabetes is a long process, has different types of pathological changes, and is changeable. The symptoms of different types, such as excessive drinking, middle elimination, diaphragm elimination, and elimination of spleen and gallbladder, show a complex process of DM, and the prognosis lies in complications [20, 21]. In the current textbook of Internal Medicine of TCM, Xiao Ke Pian continues, enriches, and develops the theories of “overflow,” “elimination,” and “digestion” in the Internal Classic, puts forward the classification of upper, middle, and lower elimination, and increases the sweet content of urine [22]. Related diabetes, including western medicine type 1 and type 2 diabetes and its complications, coordinate Sanxiao and include the classification and treatment of various types of syndromes. The pathological alterations involve internal and external diseases, women, children, facial features, orthopaedics, and dermatology. Scholars proposed that “DN can be regarded as an inflammatory disease induced by metabolic disorders” [23]. On the other hand, the theory, nature, characteristics, and essence of the disease of eliminating thirst in TCM are highly summarized as “deficiency of Wei qi, exhaustion of camp qi” and “struggle between numbers.” The argument includes the content of DN and meets the risk factors of metabolic disorder of sugar, fat, lipids, and proteins, leading to deep tissue, viscera, blood stasis, and the theory of occurrence of DN. The essence of diabetes may be understood as the metabolic disorder of Ying Qi and the immune function of Wei Qi, the blood is the host, the related tissues and organs are obstructed and damaged, and subtle leakage is difficult to heal [24]. Clinically, no matter the different complications of diabetes, how the condition evolves, and the existence of metabolic disorders of sugar, lipid, and protein, it is not eliminated because of the occurrence of nephropathy but reflects further deterioration and is not cured. The importance and difficulty of its prevention and treatment reflect the correct scientific conclusion of “no treatment of one's own disease, no treatment of one's own disease, no treatment of chaos, and no treatment of chaos” in Neijing [25].

The dominant disease of TCM means that there is no good treatment method or curative effect in western medicine at present, but TCM can be treated with a definite curative effect, or the curative effect of traditional Chinese and western medicine is definite, but the adverse reactions of TCM are relatively few, which is not easy to bring about drug-induced and iatrogenic diseases [26–28]. TCM has many advantages in the treatment of “eliminating thirst nephropathy,” which has been continuously optimized on the basis of summing up clinical experience for many years. However, the condition of Xiaoke nephropathy is complicated, and the syndrome differentiation of Zang-fu organs is difficult to cover all syndrome types. According to the syndrome differentiation of the six meridians, the location of the disease is determined by three yins and three yangs, clear disease, taking into account qi, blood and body fluid, and pathological products, combined with physical differences and layers of in-depth, to analyze and summarize the various symptoms in the process of occurrence and development of the disease [29]. It includes four aspects: disease, pulse, syndrome, and treatment, and the treatment includes sweat, vomiting, lower, and eight methods of warming, clearing, eliminating, and tonifying, which are the source of many syndromes differentiation and treatment methods in later generations [29, 30]. Syndrome differentiation of the six meridians is the general outline; when the use of general syndrome differentiation cannot work, the use of syndrome differentiation of the six meridians will often get unexpected results. Therefore, we used six meridian syndrome differentiations to optimize the dominant diseases of Xiaoke nephropathy, which had been successfully verified. This study showed that compared with the two groups, the study group was significantly effective in 34 cases, effective in 12 cases, and ineffective in 4 cases, and the effective rate was 92.00%; the control group was significantly effective in 16 cases, effective in 18 cases, and ineffective in 16 cases, and the effective rate was 68.00%. The effective rate in the study group was higher compared to the control group (*P* < 0.05). In the comparison of TCM syndrome scores, there was no significant difference before treatment (*P* > 0.05). The TCM syndrome scores of the study group were lower compared to the control at 6, 12, 24, and 36 weeks of treatment (*P* < 0.05). There was no significant difference in the indexes of UTP and UACR before treatment; however, the indexes of UTP and UACR in the study group were lower compared to the control at 6 and 12 weeks after treatment. There was no significant difference in the indexes of ALB, HbA1C, and FBG before treatment, but after treatment, the indexes of ALB increased, the indexes of HbA1C and FBG decreased in both groups, and the indexes of HbA1C and FBG in the study group were lower compared to the control, while the index of ALB in the study group was higher compared to the control. The BUN and Cr in the two groups decreased, and the indexes of BUN and Cr in the study group were lower compared to the control. With regard to the treatment safety, there was no abnormality in blood, urine, stool routine, and liver and kidney function examination in the study group. No obvious adverse reactions were found in all patients. There were 1 case of abnormal liver function and 2 cases of rash in the control group (*P* > 0.05). The basic pathogenesis of DN in the six meridians syndrome differentiation is not only to improve the local symptoms but also to regulate the whole, combined with TCM smoking prescription, TCM foot bath prescription, TCM iontophoresis, acupuncture, moxibustion, acupoint application, acupoint injection, and so on. Through direct contact with the skin, dispelling cold and dredging collaterals relieve pain, improve local circulation, further improve local symptoms, and indirectly reduce blood sugar through overall regulation. Of note, to restore the damaged renal function to the nourishment of essence, blood, and body fluid and to include the characteristic nursing of TCM, the clinical curative effect has been significantly improved under a multipronged approach. This study may also have disadvantages such as poor sample representation, inappropriate control selection, and bias in recall of exposure history. However, we tried our best to avoid them during the study to obtain reliable results.

In conclusion, the optimized scheme of comprehensive treatment of TCM under the guidance of classical theory in the treatment of DN may be through the improvement of metabolic disorders, angiopathy, neurotrophic disorders, antioxidant stress, and other ways, multilinks and multitargets, to repair nerve damage, improve renal function, improve patients' TCM syndromes, signs, and changes of various indicators, and delay the progress of the disease.

## Figures and Tables

**Figure 1:** Comparison of UPT and UACR indexes between two groups of patients.

**Figure 2:** Comparison of ALB, HbA1C, and FBG indexes between two groups of patients.

**Figure 3:** Comparison of BUN and Cr indexes between two groups of patients.

**Table 1:** Comparison of the curative effect (*n*/%).

Group	*N*	Significant effect	Effective	Invalid	Efficiency
C group	50	16 (32.00)	18 (36.00)	16 (32.00)	34 (68.00)
R group	50	34 (68.00)	12 (24.00)	4 (8.00)	46 (92.00)
*χ* ^2^					9.000
*P*					<0.001

**Table 2:** Comparison of TCM syndrome scores ($\bar{x}\pm s$, points).

Group	*N*	Before treatment	Treatment for 6 weeks	Treatment for 12 weeks	Treatment for 24 weeks	Treatment for 36 weeks
C group	50	24.84 ± 2.34	23.67 ± 2.41	21.49 ± 1.22	19.93 ± 3.31	14.49 ± 3.55
R group	50	24.59 ± 2.45	21.56 ± 2.55	18.69 ± 2.34	16.31 ± 4.21	10.48 ± 1.56
*t*		0.521	4.252	7.502	4.779	7.312
*P*		>0.05	<0.01	<0.01	<0.01	<0.01

## Data Availability

No data were used to support this study.
